# Research on Domain-Specific Knowledge Graph Based on the RoBERTa-wwm-ext Pretraining Model

**DOI:** 10.1155/2022/8656013

**Published:** 2022-10-12

**Authors:** Xingli Liu, Wei Zhao, Haiqun Ma

**Affiliations:** ^1^School of Computer Science and Technology, Heilongjiang University of Science and Technology, Harbin 150020, Heilongjiang, China; ^2^School of Information Management, Heilongjiang University, Harbin 150080, Heilongjiang, China

## Abstract

The purpose of this study is to solve the effective way of domain-specific knowledge graph construction from information to knowledge. We propose the deep learning algorithm to extract entities and relationship from open-source intelligence by the RoBERTa-wwm-ext pretraining model and a knowledge fusion framework based on the longest common attribute entity alignment technology and bring in different text similarity algorithms and classification algorithms for verification. The experimental research showed that the named entity recognition model using the RoBERTa-wwm-ext pretrained model achieves the best results in terms of recall rate and F1 value, first, and the F value of RoBERTa-wwm-ext + BiLSTM + CRF reached up to 83.07%. Second, the RoBERTa-wwm-ext relationship extraction model has achieved the best results; compared with the relation extraction model based on recurrent neural network, it is improved by about 20%∼30%. Finally, the entity alignment algorithm based on the attribute similarity of the longest common subsequence has achieved the best results on the whole. The findings of this study provide an effective way to complete knowledge graph construction in domain-specific texts. The research serves as a first step for future research, for example, domain-specific intelligent Q&A.

## 1. Introduction

With the advent of the big data era and artificial intelligence, the knowledge graph in the domain-specific application has received widespread attention. Knowledge map is a new concept proposed by Google in 2012, which is essentially the knowledge base of semantic network. As an effective knowledge representation method of cognitive intelligence of the new generation of artificial intelligence, knowledge graph uses open-source information to train cognitive models and then applies this model for cognitive application, which is an effective formation of anthropomorphic thinking. It has not only become the most intuitive and understandable framework for knowledge representation and reasoning but also improved the efficient of knowledge discovery, such as the problem system based on the domain-specific knowledge graph. However, when the knowledge graph is successfully applied in many fields, ambiguity, difficult links, data sparsity in special fields, and other problems hinder the application task effect based on the domain-specific knowledge graph. Especially in some fields with complex data sources and limited available data, how to provide an accurate knowledge extraction model for new knowledge cognition according to the needs of the field and, at the same time, how to effectively link and fuse the discovered new knowledge with the knowledge base or how to effectively link and fuse the multisource heterogeneous data with the knowledge base is an important foundation for the application of knowledge maps in some fields at present. In view of this, since open-source intelligence such as military books and the Internet has been used as the data source to solve related problems such as the automatic construction of the domain-specific knowledge graph, this research serves as a first step for future research, for example, the construction of knowledge graphs Q&A application. The innovative contribution of this research is as follows:

1. The RoBERTa-wwm-ext model is used to enhance the knowledge of the data in the knowledge extraction process to complete the knowledge extraction including entity and relationship
2. This study proposes a knowledge fusion framework based on the longest common attribute entity alignment technology and brings in different text similarity algorithms and classification algorithms for verification, all of which have achieved good results

## 2. Related Work

The knowledge graph was proposed by Google in 2012, and its essence is a semantic network knowledge base. The knowledge graph is divided into a general knowledge graph and a domain-specific knowledge graph. For the former, it emphasizes the scope of knowledge, while for the latter, it emphasizes the accuracy of domain-specific knowledge. At present, the construction and exploration technology of knowledge graphs at home and abroad has become mature. Many research institutions have successively created some large-scale general knowledge graphs, such as YAGO [1], Wikidata [2], and DBpedia [3]. However, for knowledge graphs in professional fields, the services it provides for people are still far from meeting the needs. For this reason, academia and industry have paid more attention to the research of domain-specific knowledge graphs with high professional knowledge accuracy.

Due to the sensitivity of data and low resource information in the field of military security, knowledge graph research in this field is relatively lacking, and the research progress is slow. F. Liao et al. [4], using the knowledge extraction method based on the BiLSTM model, studied the knowledge graph construction of the US military equipment and designed and implemented the US military equipment knowledge graph system. C. Liu et al. [5], aiming at the problems of loose structure of the military equipment database, difficulty in using effectively, low storage efficiency, and chaotic management, used the entity relation extraction method of the dependency syntax tree and CRF to extract information from unstructured text data, build a knowledge map of the military equipment, and achieve good results. D. Song et al. [6] proposed a military knowledge graph construction method based on bibliographic data of military disciplines to solve the problems of sparse data distribution, weak data correlation, and difficulty in using data effectively in the retrieval process of military industrial academic research content. This method designs the structure of the knowledge graph according to the bibliographic information characteristics of the article and uses the information-rich article titles and keywords to study entity extraction, entity classification, knowledge graph storage, and visualization. Yao Yi et al. [7] relied on the structured data of the existing arsenal to build the equipment concept map, using the method of iterative learning, based on open multisource data to complete the equipment entity to ensure the breadth and depth of the concept map precision. Xing Meng et al. [8] proposed a technical framework for the construction and application of knowledge graphs in the military domain regarding the opportunities and challenges currently faced by knowledge graphs in the military domain. It also discusses the key issues and core technologies in all aspects of the knowledge life cycle, such as knowledge representation based on the ontology system, knowledge extraction based on machine learning, cross-domain-specific knowledge fusion, knowledge computing, and knowledge application. Zhao Yu et al. [9] used the BiLSTM + CRF model for military named entity recognition, extracted relation words through syntactic analysis and hierarchical Dirichlet process (HDP) clustering, and obtained entities and the relationships between entities to build a military knowledge graph.

Knowledge fusion is an important link in the process of domain-specific knowledge graph construction and an important means to ensure knowledge quality and knowledge update. At present, in the process of knowledge graph research in the military field, the technology for knowledge fusion is relatively lacking. In the general field, knowledge fusion is usually based on cross-language entity alignment and same-language knowledge base entity alignment technology research. Cross-language entity alignment techniques mainly include representation learning methods based on translation models and graph neural networks. The translation model takes TransE [10] as the basic model. Models such as JE [11], MTransE [12], IPTransE [13], and AttrE [14] have improved it by using methods such as attribute, relation information, and iterative training and obtained a good effect. The graph neural network uses the global structural information of the graph to match the entities to be aligned in the two knowledge graphs. The GCN-Align [15] model is an earlier model that uses a graph neural network algorithm for entity alignment. It proposes a cross-language knowledge graph alignment method based on a graph convolutional network. The research on entity alignment of the same language is based on the Chinese heterogeneous encyclopedia knowledge base and adopts the paired entity alignment technology with the text similarity algorithm as the core.

It can be seen from the above that most of the knowledge graphs in the military field focus on the construction of knowledge graphs of weapons and equipment. Some military knowledge graph research does not subdivide the ontology granularity and builds a military knowledge graph equivalent to an encyclopedia, which is similar to the military module in the general knowledge graph and cannot meet accurate knowledge services. At present, the only research on knowledge graph construction in the military field mainly focuses on the extraction of knowledge, and there are relatively few studies on knowledge fusion. Based on the research on the military intelligence information of major military news platforms and the suggestions of military experts, this study refines the data granularity of the knowledge graph in the military field and extracts open-source military information through the deep learning technology. Second, this study obtains the diverse and heterogeneous military domain knowledge base on the Internet, combines text similarity and machine learning algorithm, proposes a knowledge fusion algorithm framework based on the longest common attribute entity alignment technology, which is used for knowledge fusion and updating, and then, constructs a high-quality maintainable knowledge graph of the military.

## 3. Key Technology

The construction of the domain-specific knowledge graph is divided into the construction of the ontology layer and the data layer. In this article, by studying the influence of data distribution and data granularity in the open-source military intelligence on the quality of knowledge graph construction, the ontology of the graph is divided into 9 entity types, including countries, aircraft carriers, missiles, radars, ships, aircraft, military bases, waters, and islands, and the relationship is divided into 5 types: country, collaboration, activity, equipment, and NULL, which are used to verify the reliability of the knowledge graph construction experiment. The definition of the relationship between entities is shown in Table 1.

The technologies of domain-specific knowledge graph data layer construction mainly include domain-specific data acquisition, knowledge extraction, knowledge fusion, knowledge storage, and graph visualization. Among them, knowledge extraction and knowledge fusion technology are the most reused, which determine the efficiency and quality of graph construction. Therefore, this study focuses on knowledge extraction and knowledge fusion technology in the construction of a knowledge graph. The technical architecture of the knowledge graph construction is shown in Figure 1.

### 3.1. Data Preprocessing

#### 3.1.1. Data Collection

The knowledge extraction module of this study takes the military intelligence information data as the main research object, and the data mainly come from open-source military news. Crawler technology is used to collect unstructured text information in the global military, military forums, and military modules in various news platforms.

The external knowledge base in the knowledge fusion module of this study mainly comes from two aspects. On the one hand, it is to obtain existing external knowledge bases. For example, data in the open-source weapon and equipment knowledge graph (OpenKG.CN) and the US military knowledge base data (Heilongjiang University of Science and Technology Cognitive Intelligence Experiment) provide existing structured knowledge bases. On the other hand, crawler technology is used to crawl semistructured military data in the open-source encyclopedias, such as Weapon Encyclopedia (http://www.wuqibaike.com/) and Wikipedia.

#### 3.1.2. Data Annotation

Data annotation is an important part of data preprocessing, which determines the quality of knowledge extraction. The entity annotation adopts the BIO annotation method; that is, the “B-entity type” indicates the mark of the beginning word of the entity, the “I-entity type” indicates the mark of the subsequent word of the entity, and “O” indicates the nonentity part. According to the definition of the ontology library, this study annotates 9 types of military entities, including NAT (country), PLA (aircraft), VES (ship), MIS (missile), WAT (water area), AIR (aircraft carrier), BAS (military base), RAD (radar), and ISL (island). An example of entity annotation is shown in Figure 2.

Relation annotation is based on entity annotation. We segment the text data with entity annotations in units of sentences and judge and annotate the relationship between entities contained in each unit according to the definition of the relational ontology library. Examples of relational annotations are shown in Table 2.

### 3.2. Knowledge Extraction

Knowledge extraction is an important step in the process of knowledge graph construction, which is mainly divided into two parts: namedentity recognition (entity extraction) and relation extraction. In this study, the method based on deep learning is used to extract knowledge from unstructured text data, and the related structured knowledge base is extracted according to the organizational structure design rules of the knowledge base. This article mainly studies knowledge extraction from unstructured text data and uses a pretraining model to vectorize text data to enhance knowledge. The acquired text semantic feature vector is combined with the deep learning model to learn the features of a large number of texts corpus and realize the knowledge extraction of unstructured text data.

#### 3.2.1. RoBERTa-wwm-ext Pretraining Model

The BERT [16] (Bidirectional Encoder Representation from Transformers) model is a pretraining model for encoding text characters proposed by Google in 2018, which uses the idea of transfer learning. Knowledge or patterns learned in one domain or task are applied to a different but related domain or problem. The BERT model mainly uses the encoder structure of the transformer model [17], which can better obtain the semantic relationship in the text data. The BERT model uses massive Wikipedia data for model training so that each word can obtain a better vector feature.

The RoBERTa [18] (robustly optimized BERT approach) model is an improved version of the BERT model, using more training data and improving the training method. In terms of training method, RoBERTa removes the NSP (Next Sentence Prediction) task, and at the same time, compared with BERT's static masking mechanism, RoBERTa uses a dynamic masking mechanism. Although RoBERTa has only slightly improved the model mechanism, it has achieved an effective improvement in the use effect.

WWM [19] (Whole Word Masking) is the whole word mask, which changes the method of using a single Chinese character as the unit of mask in the Chinese BERT model to mask the whole Chinese word. The advantage of such training is that the words encoded by the model have the meaning of the context words.

The Harbin Institute of Technology iFLYTEK Joint Laboratory released the Chinese RoBERTa-wwm-ext pretraining model, which achieved the best results in several natural language processing tasks. Therefore, this study uses the RoBERTa-wwm-ext pretraining model open sourced by the Harbin Institute of Technology to obtain text vectors with semantic features and encode the text.

#### 3.2.2. Named Entity Recognition Model

The named entity recognition model in this study is mainly divided into three layers, namely, the text encoding layer of the pretraining model, the bidirectional long short-term memory network layer (BiLSTM), and the conditional random field layer (CRF). The structure of the model is shown in Figure 3.

First, this model uses sentences containing military information as input data and encodes the text information of the sentences through the RoBERTa-wwm-ext model. A sequence of word vectors (*X*_1_, *X*_2_, ⋯,*X*_*n*_) with semantic information is obtained and fed into a bidirectional LSTM layer to automatically extract the features of sentences. The bidirectional LSTM layer splices the hidden state sequence (*h*_1_, *h*_2_, ⋯, *h*_*n*_) output by the forward LSTM and the sequence output by the reverse LSTM at the corresponding position according to the position, accesses the linear layer, and maps it into a *K*-dimensional hidden vector. Among them, *K* is the number of entity labels. At this time, *K* classification can be performed on the *P* vector corresponding to each character vector, and data labeling can be performed. To better obtain sentence-level annotation information, the output *P* vector is input into the CRF layer.

#### 3.2.3. Relation Extraction Model

The relation extraction model consists of a text encoding layer, a fully connected layer, and a multiclassifier layer. First, we obtain entity A and entity B whose relationship needs to be determined in the text data and the text data containing these two entities and connect the three to form the input text of the model. The text encoding layer encodes the input text data to form a hidden layer state vector with semantic features. The fully connected layer is used to normalize the obtained feature vector containing semantics, and the classification result is input through the multiclassifier layer. It is expressed in a mathematical equation as follows:

(1) $$\begin{array}{c} H={RoBETa}_{wwm}\left[concat\left(entA+entB\right)+txt\right]\text{,}\\ h=wH+b,p=softmax\left(h\right)\text{,} \end{array}$$

where *H* represents the semantic feature vector of the hidden layer obtained by the RoBERTa-wwm-ext model, *h* is the output of the fully connected layer, *w* and *b* are the weight and bias parameters, respectively, and *p* is the input probability of each relation label. The model structure is shown in Figure 4.

### 3.3. Knowledge Fusion

The knowledge obtained through knowledge extraction has a wide range of sources, the quality of knowledge from different sources is different, and the expression form is not uniform, which will lead to problems such as knowledge redundancy and low accuracy. Integrating multisource and heterogeneous knowledge and solving problems such as knowledge duplication is the key to improving the quality of knowledge graph construction. First, knowledge fusion is to fuse entities with different expressions of the same entity concept from multiple data sources to obtain unified knowledge. Knowledge fusion is divided into two stages. In the first stage, knowledge fusion is performed on the extracted results to ensure the formation of high-quality knowledge graphs. In the second stage, based on the constructed knowledge graph, knowledge fusion is carried out with the external knowledge base to realize the expansion and update of knowledge.

#### 3.3.1. Knowledge Fusion Framework

The knowledge fusion architecture of this study is shown in Figure 5. The data come from two parts, namely, the result of knowledge extraction and the external knowledge base, corresponding to two stages of knowledge fusion. The data preprocessing process organizes the structured and semistructured data in the external knowledge base into unified knowledge triples, through manual ontology matching and entity classification and entity alignment within each ontology type, and finally completes knowledge fusion.

#### 3.3.2. Entity Alignment

The entity alignment algorithm is the core of the knowledge fusion framework. This study adopts the paired entity alignment algorithm; that is, the similarity screening of entities is performed in advance, the entities that cannot be similar are filtered out, and the possibly similar entities are marked as candidate entity pairs. According to the attribute similarity between candidate entity pairs, a machine learning algorithm is used to classify them into a matching set or a nonmatching set. The algorithm flow is shown in Figure 6.

The attribute similarity algorithm is an important part of the paired entity alignment algorithm in this study. Due to the different sources of knowledge, the attribute lengths of entities describing knowledge are inconsistent. Therefore, this study proposes a method of maximum common attribute length to calculate the similarity of attributes. We select the attribute of the maximum coincidence of two entities in the entity pair to calculate, which is expressed as follows:

(2) $$\begin{array}{c} CommomPropertty\left(e_{1},e_{2}\right)={Property}_{e_{1}}\cap {Property}_{e_{2}}\text{.} \end{array}$$

Among them, *e*_1_ and *e*_2_ represent entities and Property_*e*_1__ and Property_*e*_2__ represent attributes corresponding to entities. The lengths of common attributes between different entity pairs are inconsistent, which leads to unequal lengths of attribute similarity feature vectors obtained from attribute similarity calculation. Therefore, the obtained feature vector is subjected to dimension reduction and normalization processing. Since the name of the entity has a high degree of identification for the entity, the entity name is used as the main attribute Property_main_, and the other attributes are used as auxiliary attributes Property_secondary_ = {*P*_*s*1_, *P*_*s*2_, ⋯, *P*_*s*_}. The auxiliary attributes are averaged to reduce the original multidimensional feature vector to two dimensions. Thereby, the similar feature quantities of the attributes can be unified. Normalizing the attribute similarity vector can represent the similarity between entity pairs. Based on the abovementioned ideas, the similarity between entity pairs can be expressed as follows:

(3) $$\begin{array}{c} {sim}_{Propertty\left(e_{1},e_{2}\right)}=\left\{sim\left({Property}_{main}\right),ave\left[sim\left({Property}_{secondary}\right)\right]\right\}\text{,}\\ ave\left[sim\left({Property}_{secondary}\right)\right]=\frac{\sum_{i}^{N}sim\left(p_{si}\right)}{N},N=\left|{Property}_{e_{1}}\cap {Property}_{e_{2}}\right|\text{.} \end{array}$$

The attribute similarity algorithm adopts text similarity algorithms such as SimHash [20], edit distance, longest common subsequence, and BERT word embedding. The classification algorithm adopts machine learning algorithms such as support vector machine [21] (SVM), decision tree, logistic regression, and naive Bayes. Combined experiments with different attribute similarity algorithms and classification algorithms are used to verify the effectiveness of entity alignment.

## 4. Experiments

### 4.1. Datasets

This study takes the military intelligence information data as the main research object, and the data mainly come from open-source military news. We use crawler technology to collect unstructured text information containing the military intelligence information such as global military, military forums, and military modules in various news platforms for knowledge extraction. Second, we extract the structured and semistructured data in the open-source weapon and equipment knowledge graph, weapon encyclopedia, Wikipedia knowledge base, and the US military knowledge base for knowledge fusion. The experimental datasets in this study are divided into three parts: named entity recognition, relation extraction, and entity alignment.

#### 4.1.1. Named Entity Recognition Dataset

The named entity recognition part of the dataset in this study is constructed by manual annotation. The dataset contains 9 types of entity labels, including a total of 53,295 entity labels and 14 MB of text data. The distribution of entity labels is shown in Table 3.

#### 4.1.2. Relation Extraction Dataset

The relation extraction part of the dataset in this study is jointly constructed by the methods of automatic labeling of entity-relationship types and manual review. The dataset contains a total of 2251 pieces of data with 5 types of relationship labels. The distribution of relationship labels is shown in Table 4.

Since the length of the text corpus has a certain influence on the difficulty of relation extraction, the text length is counted. The text length distributions of the training set and test set are the same, as shown in Figure 7.

#### 4.1.3. Entity Alignment Dataset

The data used in this study to verify the entity alignment algorithm in the knowledge fusion framework come from two data platforms, the open-source military weapon and equipment knowledge graph and the weapons encyclopedia. From the acquired data, a total of 1324 prealigned entity pairs were obtained by random sampling and manual alignment of four types of data, including missile weapons, aircraft carriers, vessels, and plane. These entity pairs contain a total of 28447 attribute triples. The specific data distribution is shown in Table 5.

Through the analysis of the dataset composed of two data sources, it is found that two entities have the same name in some prealigned entity pairs. In order to improve the robustness of the trained model, a new entity name is formed by inserting, deleting, or replacing characters in the data from one of the sources according to the naming rules of the military field and forming a prealigned entity pair in this experiment. Negative samples are obtained by randomly replacing entities between prealigned entity pairs. The prealigned entities are scrambled by their data categories to form 50% positive and 50% negative samples, and finally, 2648 entity pairs are formed for alignment experiments.

### 4.2. Experimental Parameters

#### 4.2.1. Named Entity Recognition Model Parameters

The amount of data used in the training of the named entity recognition model and the parameter volume of the pretraining model are large. Considering the hardware environment of the experiment and the reliability of model training, the main parameters of the named body recognition model in this study are shown in Table 6.

#### 4.2.2. Relation Extraction Model Parameters

The size of the hidden layer state vector of relation extraction and the size of the number of hidden layers refer to the RoBERTa model parameters. Considering the distribution of text lengths in the dataset, we set the maximum text input (max_length) to 128 characters. Other parameters are based on the experience of deep learning model training, and the specific experimental parameter settings are shown in Table 7.

### 4.3. Evaluation Metrics

This experiment uses three indicators of precision, recall, and F1 value to evaluate the reliability of the model. The calculation expressions of the three indicators are as follows:

(4) $$\begin{array}{c} precision=\frac{TP}{TP+FP}\text{,}\\ recall=\frac{TP}{TP+FN},F1=\frac{2\times precision\times recall}{precision+recall}\text{,} \end{array}$$

where *TP* represents the number of labels that the model can correctly detect, *FP* represents the number of irrelevant labels detected by the model, and *FN* represents the number of labels not detected by the model.

### 4.4. Experimental Results

#### 4.4.1. Named Entity Recognition Experiment Results

The named entity recognition dataset is used for data, the size of the training dataset is 10.3 MB, and the test is 3.2 MB. The experimental results of the trained model on the test set are shown in Table 8. The accuracy of some of the entity labels is low, the reason is that the amount of labeled data for this part of the entity labels is small, and the number of occurrences in the military dataset used in this experiment is small. However, it does not affect the reliability of the model and can be corrected by increasing the number of corresponding labels.

To verify the effectiveness of the named entity recognition model and dataset, four groups of comparative experiments were set up in this experiment as shown in Table 9. These include the BiLSTM + CRF model, IDCCN model, BERT + BiLSTM + CRF model, and BERT-wmm-ext + BiLSTM + CRF model. From the results of the comparative experiments, it can be seen that the named entity recognition model using the RoBERTa-wwm-ext pretrained model achieves the best results in terms of recall rate and F1 value.

#### 4.4.2. Relation Extraction Experiment Results

The relation extraction experiment uses 1800 text data for model training and 451 text data for testing. Each relationship label has achieved better results on the test set, and the experimental results of the trained model on the test set are shown in Table 10.

To verify the effectiveness of the relation extraction model and dataset, four groups of comparative experiments were set up in this experiment, and the more popular deep learning models were selected as comparative experiments. The comparative experimental results are shown in Table 11. From the comparative experimental results, it can be seen that the BERT series of relationship extraction models have good results, and the BERT-wwm-ext relationship extraction model has achieved the best results, which is similar to the RoBERTa-wwm-ext-based relationship extraction model used in this study. Compared with the relation extraction model based on recurrent neural network, it is improved by about 20%∼30%.

After further analysis, there are two reasons for the excellent effect of the experiment. On the one hand, it is the superiority of the BERT model, which is formed based on massive data training and has a good ability to express knowledge. The RoBERTa-wwm-ext model is a further improvement of the BERT model, so the experiment has achieved good results. On the other hand, the dataset used for the experiment contains fewer relationship types, which may lead to a high effect on the experiment. In the future, the relationship type of the dataset will be increased to further verify the effect of the model.

#### 4.4.3. Entity Alignment Experiment Results

The entity alignment experiment in this study is based on the scikit-learn and bert4keras framework. Combined experimental analysis of four attribute similarity algorithms of SimHash, edit distance, longest common subsequence (LCS), and BERT word embedding and four classification algorithms of support vector machine (SVM), decision tree, logistic regression (LR), and naive Bayes (NB) was conducted. The experimental results are shown in Table 12.

According to Table 12, the entity alignment algorithm based on the attribute similarity of the longest common subsequence has achieved the best results on the whole, and the combination with the classification algorithm of logistic regression has achieved the best results. Second, the algorithm based on SimHash is better overall and achieves the local optimum when combined with the decision tree classification algorithm.

## 5. Discussion

This study aims to provide an efficient and reliable method for the construction of knowledge graphs in specific fields. Taking the military field as an example, the two modules of knowledge extraction and knowledge fusion mentioned in the study are experimentally verified. Different from previous studies, this study uses the pretrained model RoBERTa-wwm-ext for knowledge enhancement, which improves the effect of knowledge extraction. In addition, this article studies the knowledge fusion module that is less studied in the construction of domain knowledge graphs in the past and proposes a knowledge fusion framework based on the longest common attribute entity alignment technology. In the process of graph construction, it is used to ensure its quality, and it is used for knowledge expansion and update in the process of graph maintenance.

In the knowledge extraction module, this study uses the RoBERTa-wwm-ext model to vectorize text data, which is different from the previous random initialization or word2vec for text vectorization. The advantage of this is that the vector of the knowledge extraction model in the data input stage has excellent semantic expression ability, so the effect of the trained knowledge extraction model will be greatly improved. Most of the previous research on domain knowledge graph construction focused on knowledge extraction, but this research not only studies knowledge extraction but also studies knowledge fusion and proposes a knowledge fusion framework. The framework brings in different text similarity algorithms and machine learning classification algorithms, all of which have achieved good results.

There are also some limitations in this study. First, this study uses the manual annotation method in the data preprocessing stage to annotate the named body recognition dataset and relation extraction dataset, which increases a lot of labor costs. Although the most effective method is manual annotation at present, semiautomatic annotation methods will be considered in the future, for example, annotating a small number of correct seed data and using the seed data to iteratively annotate most of the data.

Second, in the knowledge extraction stage of this study, the recognition effect of some entity labels in the named entity recognition experiment is not good. After analyzing the experimental process, in the named entity recognition experiment, due to the small number of annotations for some labels, the data distribution of each label in the data samples used for training is unbalanced, resulting in poor recognition of some labels. In the future, we will continue to optimize the datasets of each experimental module to improve the experimental effect of each module.

Third, in the knowledge fusion stage, a large amount of text similarity between entity attributes needs to be calculated in the process of entity alignment, which will inevitably lead to the low computational efficiency of the knowledge fusion framework. In the future, the domain synonym dictionary and stop word dictionary will be added to the text similarity calculation process, which can reduce the number of text similarity calculations and optimize the efficiency of the knowledge fusion framework.

## 6. Conclusion

This study combines the machine learning and deep learning technology to study the automatic construction technology of knowledge graphs in the military domain and focuses on the knowledge extraction and knowledge fusion technology in the process of domain-specific graph construction. The RoBERTa-wwm-ext model is used to enhance the knowledge of the data in the knowledge extraction process to complete the knowledge extraction. Second, this study proposes a knowledge fusion framework based on the longest common attribute entity alignment technology and brings in different text similarity algorithms and classification algorithms for verification, all of which have achieved good results. The recognition effect of some labels in the named entity recognition model in this study is not good. In the future, the model training dataset and the architecture of the model will be improved to improve the effect of entity extraction. In knowledge fusion, a large amount of data calculation needs to be performed. The current knowledge fusion framework has low computational efficiency. In the future, a domain synonym dictionary and a stop word dictionary will be added to perform word segmentation calculation on attribute information to improve computational efficiency.

## Figures and Tables

**Figure 1:** Technical architecture of knowledge graph construction.

**Figure 2:** An example of entity annotation.

**Figure 3:** The named entity recognition model.

**Figure 4:** Relation extraction model.

**Figure 5:** Framework of knowledge fusion.

**Figure 6:** Entity alignment algorithm flow.

**Figure 7:** Distribution of text length in relation extraction.

**Table 1:** Interpretation of relationship labels.

Serial number	Relation label	Relationship type interpretation
1	Country	Country to which ships, aircraft carriers, aircraft, and missiles belong
2	Collaboration	Cooperative operations among ships, aircraft carriers, and aircraft
3	Activity	Ships, aircraft carriers, and aircraft are active in a certain area target
4	Equipment	Missiles and radars equipped on ships, aircraft carriers, and aircraft
5	NULL	No relationship between entities

**Table 2:** Examples of relational annotation data.

Text	The British Royal Navy's aircraft carrier “Italia Hakujou,” the Yomikoku Navy's aircraft carrier “Satone,” and the “Soho Island” cruise ship to Dingyang completed a large-scale maritime military exercise
Entities	Aircraft carrier “Satone” and “Soho Island” cruise ship
Annotation	Collaboration

**Table 3:** Entity label distribution.

Serial number	Entity label	Number statistics
1	NAT (nation)	34833
2	PLA (plane)	8144
3	VES (vessel)	4319
4	MIS (missile)	2597
5	WAT (waters)	1351
6	AIR (aircraft carrier)	704
7	BAS (military base)	561
8	RAD (radar)	470
9	ISL (island)	316

**Table 4:** Relation label distribution.

Serial number	Relation label	Number statistics
1	Country	841
2	Collaboration	491
3	Activity	262
4	Equipment	297
5	NULL	360

**Table 5:** Distribution of prealigned entity pairs.

Label	Open-source knowledge graph (attribute triple)	Weapon encyclopedia (attribute triple)	Prealigned entity pairs
Missile weapon	3914	2641	349
Aircraft carrier	1593	1123	100
Vessel	5571	3546	360
Plane	10007	4927	515
Total	21085	12237	1324

**Table 6:** Named entity recognition model parameters.

Serial number	Parameter	Value
1	Epochs	50
2	batch_size	64
3	lstm_dim	200
4	max_seq_len	128
5	Learning rate	0.001
6	Dropout	0.5

**Table 7:** Relation extraction model parameters.

Serial number	Parameter	Value
1	Epochs	50
2	batch_size	50
3	hidden_size	768
5	max_length	128
6	Learning rate	0.001
7	Dropout	0.1

**Table 8:** Named entity model recognition results.

Label	Precision (%)	Recall (%)	F1	Number statistics
NAT (nation)	85.87	93.83	89.68	8453
PLA (plane)	79.05	76.12	77.55	1532
VES (vessel)	66.71	69.49	68.07	775
MIS (missile)	61.60	50.10	55.26	388
WAT (waters)	58.33	69.72	63.52	300
AIR (aircraft carrier)	63.64	52.34	57.44	88
BAS (military base)	50.51	48.54	49.50	99
RAD (radar)	72.46	37.88	49.75	69
ISL (island)	60.92	64.63	62.72	87
Overall	81.11	85.13	83.07	11722

**Table 9:** Comparative experimental results of named entity recognition.

Model	Precision (%)	Recall (%)	F1
RoBERTa-wwm-ext + BiLSTM + CRF	81.11	85.13	83.07
BiLSTM + CRF	81.51	84.63	83.04
BERT-wmm-ext + BiLSTM + CRF	80.96	84.90	82.89
BERT + BiLSTM + CRF	81.93	84.01	82.96
IDCNN	79.46	84.73	82.01

**Table 10:** Test results of the relation extraction model.

Label	Precision (%)	Recall (%)	F1	Number statistics
Country	99.36	96.89	98.11	161
Activity	95.00	100	97.43	57
Equipment	96.61	95.00	98.45	60
Collaboration	96.94	100	98.07	95
NULL	98.70	97.44	98.07	78
Overall	97.32	97.87	97.57	451

**Table 11:** Comparative experimental results of relation extraction.

Model	Precision (%)	Recall (%)	F1
RoBERTa-wwm-ext	97.32	97.87	97.57
BERT	96.46	96.56	96.50
BERT-wwm-ext	98.11	98.14	98.13
BiGRU-ATT	77.87	74.22	75.74
BiLSTM-ATT	68.36	66.61	67.47

**Table 12:** Comparison of the experimental results of entity alignment.

Similarity	Classification	Precision (%)	Recall (%)	F1
SimHash	SVM	97.79	97.66	97.72
SimHash	Decision tree	98.31	98.28	98.29
SimHash	LR	97.79	97.66	97.72
SimHash	NB	98.00	97.84	97.91
Edit distance	SVM	97.58	97.49	97.53
Edit distance	Decision tree	97.24	97.08	97.15
Edit distance	LR	97.37	97.31	97.34
Edit distance	NB	95.40	95.65	95.46
LCS	SVM	99.27	99.21	99.24
LCS	Decision tree	99.59	99.65	99.62
LCS	LR	99.80	99.81	99.81
LCS	NB	99.27	99.21	99.24
Word embedding	SVM	82.75	80.17	80.46
Word embedding	Decision tree	92.41	92.40	92.41
Word embedding	LR	91.47	91.44	91.45
Word embedding	NB	67.02	63.40	59.84

## Data Availability

The data supporting the findings of this study are available within the article.
